The article "Cloud-Based IoE Enabled an Urban Flooding Surveillance System" was published in 2022. Journal: Comput Intell Neurosci.

# Cloud-Based IoE Enabled an Urban Flooding Surveillance System

**DOI:** 10.1155/2022/8470496

**Published:** 2022-05-25

**Authors:** R. Dhaya, Tariq Ahamed Ahanger, G. R. Asha, Emad A. Ahmed, Vikas Tripathi, R. Kanthavel, Henry Kwame Atiglah

**Affiliations:** ^1^Department of Computer Science, College of Arts and Science-Sarat Abidha, King Khalid University, Abha, Saudi Arabia; ^2^College of Computer Engineering and Sciences, Prince Sattam Bin Abdulaziz University, Al-Kharj, Saudi Arabia; ^3^Department of Computer Science & Engineering, B.M.S. College of Engineering, Bangalore, Bull Temple Rd, Basavanagudi, Bengaluru, Karnataka-560019, India; ^4^Department of Computer Science, Faculty of Computers and Information, South Valley University, Qena, Egypt; ^5^Department of Computer Science & Engineering, Graphic Era Deemed to Be University, Dehradun, Uttarakhand, India; ^6^Department of Computer Engineering, College of Computer Science, King Khalid University, Abha, Saudi Arabia; ^7^Department of Electrical & Electronics Engineering, Tamale Technical University, Tamale, Ghana

## Abstract

A flood is defined as a surplus of water or sludge on parched soil, and a flood has originated through the runoff of water inside the water route from the various water sources like canals, etc. Intense rainfall, deforestation, urbanization, deprived water and sewerage administration, and lack of concentration toward the environment of the hydrological scheme have been the causes of urban flooding. In addition, there is a deficiency in flood assessment due to the impediment in getting data on floods to the control room from the flood-affected area. To diminish the possessions due to flooding, there ought to be an immediate move of captured statistics as of the hectic region en route to the observation room with no further wait for a completely fledged technique in the wireless settings data from the Internet of Things (IoT). The Internet of Everything (IoE) is a concept that extends the Internet of Things. In view of the fact that the wireless nodes are changeable in their environment, those effects lead to unsteadiness and uncertainty in information distribution. Therefore, there is a requirement for flood-predictable region data that may be exaggerated between the source and the control room. In the past, there were a lot of techniques set up and put into practice intended for keeping an eye on the flood spots. However, one of the biggest challenges is to have data sharing without delay and loss of data among source and destination nodes. In addition to that, the video quality also needs to be taken into consideration at the same time in receipt, as it is a tough task to determine and preplan the flood happenings completely from the normal disaster that makes scientific complicatedness more than the information being received in a wireless ad-hoc environment using IoT-based sensors. Considering all the abovementioned reasons, the proposed work comprises of three folded goals, namely, the design of a mobile ad-hoc flooding environment, the development of an urban flood high definition video surveillance system using IoT-based sensors, and experimental work on simulation.

## 1. Introduction

With the increasing intensity of weather conditions, the occurrence and harshness of urban flood events have increased globally. Floods have been the most universal and distressing of all adverse effects. The frightening number of casualties due to floods and the increasing monetary suffering annually calls for an enhanced response to flood threats [1]. Flooding causes instant damage. Lives are lost, property is ruined, and crops are destroyed in rural areas. Floods cause significant damage, interrupt economic operations, and result in food scarcity. Exploring the images from the camera and gathered data, the IoT system is able to get better supervision of floods. With the help of IoT, early flood detection can be done, which maintains a secure look in excess of a variety of normal features to envisage a flood as a caution to reduce the harm [2]. The intention of using IoT is to detect the level of water in riverbeds and determine if they are in good condition. If they go over the limit, it sends out signals and sounds an alarm to inform people. It also sends out SMS and e-mail alerts when the water level rises above the set limit. Natural failure, similar to an overflow, can overwhelm the most valuable possessions, injuring and killing people [3]. To get rid of or diminish the contact of the flood, the system should use a range of ordinary things to notice the flood by means of an IoT system that has Wi-Fi connectivity, so the collected statistics can be contacted from anyplace without problems [4]. The intensity and frequency of threat incidents, the extent to which the community and perhaps other critically outstanding debts are subjected to threats, and the shortcomings of the vulnerable resources that lead to distress harm when confronted with various hazards, all contribute to the hazard threat [5]. Since both the hotspots and the DRI studies are focused on the same hazard probabilistic principle, the results are similar [6].To become aware of a flood, the system must watch a choice of natural factors, which comprise humidity, temperature, water level, and flow level. To gather information to talk about expected issues, the system has many sensors which accumulate information for other limitations [7]. Temperature, humidity sensor, float sensor, and flow sensor with an advanced sensor module to detect the temperature, humidity, and water level. Several techniques have been measured by different writers, and most groundwater tracking algorithms produce better levels of accuracy, leading to tests that are not dissimilar in methodology and auxiliary information utilized [8]. The surveillance system also has an ultrasonic sensor mechanism that uses ultrasonic waves to determine the distance of an object from the sensor [9]. Out of these features available in any smart surveillance system, the paramount challenge is the reachability of captured images and videos to the control node or server concurrently. In addition to that, in any situation during inclement weather, the videos must reach the server amid network failure or path failure, and hence these issues are to be met properly in order to ensure that the flood monitoring with high definition videos is effectively used [10]. Multihoming requires different sets of IP addresses to be bound between the transmitter and the receiver at the same time. The retrieval of the initial transmissions at the recipient amid network model failures is one of the critical problems facing the code unit in handling the coding phase over an insecure framework such as a multihop network system [11]. Each one specifies a distinct path, and the several connections allow for simultaneous multipath data transmission for increased throughput and efficiency. Multihomed data transfer over cloud data centers is a big deal when it comes to making sure that the limited network resources needed to give a good quality of service are put in place [12]. The Internet of Things does not include anything that needs to be done by humans.

Recent studies have focused on video transmission over several interaction paths. For video distribution, concurrent multipath transmission is seen as a possible approach. The CMT method is a data transmission process in which the transmitter conveys information between two pathways over data networks at almost the same time, and the recipient may collect information from one or more outlets [13]. On the other hand, the CMT system uses the accessible network line by taking the vacant paths for transmission, which permits the transportation method to function autonomously of the essential knowledge, similar to the perception of concurrently [14]. The wireless communication network makes use of numerous system lines for improved performance and consistent access, and the best technique for distributing information traffic over several pathways is called information transportation [15]. The simple CMT, as we know, limits the total amount of information that can be transferred by limiting the length of the recipient window. Besides that, the sender attempts to enter the active route with the shortest possible transmission delay in order to send the missing packets as quickly as possible in the situation. Researchers have suggested the CMT lag is related to data reordering, but they have rarely acknowledged the common thing of data packets in strong channels [16] to keep CMT's spectrum consolidation and transmission line capabilities while increasing throughput efficiency. There are no useable partitions to choose from if the sum of continuous lost packets is too high and the total accessible partitions is less than the sum of continuous lost packets. However, the overall packet loss value cannot be used to estimate the number of continuous lost packets on a network [17]. CMT conveys data forwarding from end to end along various trails to accomplish an advanced data transmission rate in multihomed network surroundings. It is also significant to note that the parallel information transfer in heterogeneous networks might result in chunked buffers at the source and destination ends [18]. IoE is a paradigm for enhancing flood resilience by monitoring, recognizing, and reducing the undesirable and unanticipated variability induced by a critical event. The IoE is a natural progression of the IoT concept. An efficient CMT approach that maximizes real-time signal strength in distributed cloud data centers by using pathway state determination, flow rate distribution, and data transmission control. Multihomed wireless devices are becoming more efficient and widespread, allowing for spectrum aggregation for improved transmission efficiency and throughput capacity [19]. Connecting networks to increase write performance in SQL databases can be tough. IoT use cases are frequently text-intensive with unpredictable traffic surges. If your team is concerned about scalability, document databases like MongoDB or DynamoDB can be excellent solutions for handling system demand [20]. The provision of advance warning of conditions that are likely to cause flooding of property and a potential risk to life is known as “flood warning.” The primary goal of a flood warning is to save lives by giving people, their support systems, and emergency responders enough time to prepare for flooding. Thus, the objectives of this paper are as follows:

- To develop the transmission competence of flood-captured video of the monitoring surveillance system.
- To reduce the overhead of pathway switching in a multipath mobile environment during flooding.
- To reduce the amount of space in the receiver's buffer by delivering successive packets to the destination even though the packets were lost in the process.
- To be able to send out the quality description video with a multi-homed network, you need to use early warning measures.

The rest of the paper is organized as follows: Section 2 of this paper comprises the preliminary studies. The analysis on concurrent multipath wireless systems in flood monitoring is discussed in Section 3, the proposed work is described in Section 4, and the experimental results and outcomes are discussed in Section 5. Finally, the summary and conclusion are presented in Sections 6 and 7.

## 2. Preliminary Studies

This section explains the survey on various research issues and outcomes on urban flooding, high definition monitoring using a concurrent multipath wireless environment, and the role of IoT and its previous use [20]. The goal of implementing the techniques is simply to generate early warnings as natural disasters such as floods, rainstorms, tsunamis, and others that pose a major threat to life and property all over the world. It is very common for these natural threats to turn into tragedies if they are not properly monitored and taken care of [21]. This can cause financial problems, disruptions in livelihood, and damage to the town's surroundings.

The flood is the most dangerous, and its severity cannot be predicted accurately. A flood disaster can be defined as an enormous amount of water that comes suddenly and drastically upsets or hampers the normal activities of humans and animals. The worldwide outbreak of a flood can be more disturbing if these figures are combined with other copious floods at a small scale, where fewer than ten people may have died [22]. There have been a number of efforts studied internationally to increase cost-effectiveness and strengthen flood monitoring methods. Out of all the approaches, a familiar mechanism is devised with the use of computer vision, wherein pertinent images are obtained and developed to develop resolution in creating floods. These camera-based applications are cost-effective, and their wide coverage areas enable the recognition of flood levels at various points, which is better than the fixed camera sensors [23]. Computer vision is an enhanced version of an image processing technique used in all surveillance applications. It is used to enable data transmission and increase efficiency by breaking the tight bond between data streams, including their sequence numbers. The reader does not pay attention to the average packet sequence, so changing the order in the buffers is prevented [24]. The recipient must position the data received through quick pathways into its queue and check for the pending information gathered over slower pathways to be reordered for concurrent data transfer. In this example, the packets are stored in the processor buffer before being sent to the channel module to be read.

Through random linear routing protocols, the suggested methodology replaces the Internet protocol system's dependency on data packet control messages and increases throughput by removing the inherited recipient buffer limiting problem that occurs during concurrent multi-path video streaming [14]. The main challenge is exploring the correlation features of different paths, as a multipath choice must take account of the advantages of path diversity. Specific nodes or ending systems may carry out this function as the final result of the selection procedure [25]. In order to determine the condition of data packets over the path, like if they were obtained or if they were lost, the majority of the approaches are either focused on different forwarding efforts to enhance throughput or testing SCTP-CMT output in various situations with varying levels of service quality. In 2010, Xu and Wang proposed an image signal computing technique to resolve troubles like data errors in the variety of recorded moving pictures broadcast amid flood alleged regions. Transmission's channel performance tuning reliability, which accounts for performance degradation, is one of the most significant causes. In 2007, Yang et al. projected a straightforward and efficient technique for habitual tragedy discovery in floods as an early detection. In 2015, Chau Yuen et al. prepared a “Concurrent Multipath Transfer for Mobile Video Streaming-Content Aware” (CMT-CA) explanation based on the predictable captured constraints. In 2015, Jun-liang et al. planned a content-aware concurrent multipath transport designed for better-definition video streams than heterogeneous mobile systems within a parallel and disseminated scheme. In 2013, Chang Qiao Xu et al. developed a Quality-Alert adaptive simultaneous multipath information shift in heterogeneous networks, where different types of networks were used. In 2013, Scott Pudlewski et al. discussed non-linear compressed videos with high resolution encoding and wire-free transmission. In 2013, Pudlewski et al. presented a solution for assisting in streaming aligned videos without the use of modern sensors for capturing high-contrast images. In 2019, Rajendra et al. proposed centralized techniques for flood evaluation data collection. From the above study of national and international current status with regard to the flood monitoring surveillance system for HD video transmission in an ad-hoc environment, it is concluded and inferred that there is a heavy requirement for a better flood monitoring system by taking the parameters, namely, the quality of video and reliability in transmission, by reducing packet loss and delay time, and to enhance the efficiency of the flood monitoring surveillance system.

## 3. Analysis on the Concurrent Multipath Wireless System in Flood Monitoring

The key factor behind the usage of concurrent multipath is to utilize the multipath effectively in order to be away from path failure and packet loss in the most possible way [26]. The purpose of this CMT is that in the lost packets, irregular pathways can be established as quickly as possible, and it resends the lost packets speedily to keep them away from all paths from deteriorating, merely for the abnormity of a single pathway, which confines the process of the entire connection [27]. The CMT technology combines many pathways together again to leverage the network bandwidth connections for communication. It is similar to the concept of transit virtualization in that it permits transport mechanisms to operate independently of the underlying technology. The capacity of a CMT connection to provide several IP pathways to its peer terminal is known as multihoming. Multihoming associations have the advantage of being more fault-tolerant when it comes to physical network failures and other issues on the interfaces [28]. For flood monitoring surveillance systems, the need for a concurrent multipath system is needed to ensure the data's safety and reliability while transferring for the following reasons:

- They focus on getting data rather than broadcasting them and how important they are for flood management schemes.
- The high energy efficiency schemes do not work well enough to make high-quality videos because they do not use IoT-based sensors in real time.
- The earlier period records of flooding are not explained well, and the algorithms for distributing the captured pictures do not consider the status of time-varying one to decrease packet loss without delay by not occupying more bandwidth.

This method of CMT attempts to classify the packet loss [23] of different paths and then disperse data packets iteratively across several possible paths in order to mitigate variations in packet loss and enhance data transmission performance [22]. The throughput of the path Pi, denoted as TPi, can be determined as follows:

(1) $$\begin{array}{c} T_{pi}=\frac{c}{\left({\text{RTT}}_{\text{Pi}}\;\times \sqrt{{\text{PLR}}_{\text{Pi}}}\right)}, \end{array}$$

Here, *PLR*_*Pi*_ refers to the packet loss rate of the path *p*_*i*_. In many cases, the most critical factor for determining pathway performance is RTT. Moreover, an independent sample technique that calculates the RTT of any packets transmitted on every path cannot fairly reflect the RTT variation mechanism or predict the pattern of path performance variations, and *RTT*_*Pi*_ denotes the current value of the path can be considered as follows:

(2) $$\begin{array}{c} RTT=w\times RTT_{pi}+\left(1-w\right)\times \phi_{pi},\\ \text{Where},\phi_{pi}=t-T_{\text{send}}-\Delta T. \end{array}$$

*T*_send_ is the time difference used to calculate transmission time and *w* is a weighting parameter with a value of 7/8. Though this time difference denotes the time *t* at which selective acknowledgment is sent from receiver to sender. Then, *PLR*_*pi*_ can be calculated as follows:

(3) $$\begin{array}{c} PLR_{pi}={\left(\frac{c}{{\text{T}}_{\text{pi}}}\times {\text{RTT}}_{pi}\right)}^{2}. \end{array}$$

∆T denotes the time interval between each packet's arrival at the receiver process. The value of *T*_*pi*_ can be computed as follows:

(4) $$\begin{array}{c} {\text{T}}_{\text{pi}}=\frac{{\text{CWND}}_{\text{pi}}}{\left({\text{RTT}}_{\text{p min}}\right)}, \end{array}$$

where *RTT*_min_ denotes the minimum value in all paths and CWND_pi_ denotes the congestion window size of the path *p*_i_

(5) $$\begin{array}{c} {\Delta \text{PLR}}_{\text{pi}}=\frac{{\text{PLR}}_{\text{pi}}{-\text{PLR}}_{\text{pi}}{}^{\text{avg}}}{{\text{PLR}}_{\text{pi}}{}^{\text{max}}{-\text{PLR}}_{\text{pi}}{}^{\text{min}}},\\ {\text{PLR}}_{\text{pi}}{}^{\text{max}}=\frac{1}{\text{k}\left(\sum_{\text{n}=1}{\text{PLR}}^{\text{n}}{}_{\text{pi}}\right)},\\ {\text{PLR}}_{\text{pi}}{}^{\text{max}}=\text{max}\left\{{\text{PLR}}^{1}{}_{\text{pi}}{\text{,PLR}}^{2}{}_{\text{pi}}{\text{,…PLR}}^{\text{k}}{}_{\text{pi}}\right\},\\ {\text{PLR}}_{\text{pi}}{}^{\text{min}}=\text{min}\left\{{\text{PLR}}^{1}{}_{\text{pi}}{\text{,PLR}}^{2}{}_{\text{pi}}{\text{,…PLR}}^{\text{k}}{}_{\text{pi}}\right\}. \end{array}$$

As below mentioned, we can identify packet loss and improve data transmission performance for multiple paths based on *PLRP* and Δ*PLRP* by the values of *PLR*_avg_, *R*max_pi_, *PLR*min_pi_ pi in an unreliable transmission condition.

## 4. Proposed Flooding High definition Surveillance Using the Concurrent Multipath Protocol

An efficient flood video surveillance system has been projected to observe as well as review the region where flooding is believed to be occurring in the course of better recordings in wireless ad-hoc surroundings. With the help of the CMT system in multihomed mobile networks, reliable video transmission can be achieved with the lowest delay [29]. The architecture view of the proposed system is illustrated in Figure 1. The flood surveillance system comprises three key parts, namely, the UFM-HDVSS transmission part, the multihomed wireless network part, and the receiver part. With the organization of the high definition video camera, the UFM-HDVSS transmitter section processes and promotes the continuous videos to the receiver via a multihomed mobile network. Figure 1 demonstrates the structural design of the planned system [30]. Video processing is mostly used to create high-quality visible-light videos for human consumption. Many techniques for digital video processing are derived from the fundamental concepts of digital image processing. The allocation of hardware, the binding of data flow operators and outcomes to that equipment, and the suitable connectivity of the equipment to implement the data flow path are all steps in the system design. The next job is to figure out the shortest path in wireless situations in three ways:

  Case (a): The main pathway is a perfect pathway.
  Case (b): If the main path fails, the substitute path is chosen.
  Case (c): If the substitute path fails,

By acclimating in the above cases, the progressed recorded data will be thrown all the way through the multihomed mobile network. The crucial goal of scheming multihomed simultaneous systems is to make certain that the information is not lost at all because the gathered data are needed by the control room productively and consecutively using IoT-based sensors [31]. The third path, namely, the control room, is responsible for receiving the video information for further processing. The video streaming experiments are carried out by means of a bandwidth of 400 kbps to 3.2 Mbps [32].

The communication flow represented in Figure 2 for the concurrent multipath transfer protocol for flood monitoring is illustrated. The process starts with the videos being captured and then sent to the concurrent multipath network after their initial processing to reach the destination. During path detection, there are three cases that the CMT protocol provides, which are either choosing the primary path (P1) as a default selection, and if it fails, immediately selecting an alternate path (A1) is selected in order to get through the network. Again, the protocol provides the possibility to select P1 again once an A1 fails after some roundtrip time [33, 34]. As a result, the video packet could be successfully delivered to the destination or the control room without causing any delays in the remedial actions. CMT technology combines many pathways together again to leverage the network bandwidth connections for communication. It is similar to the idea of transit virtualization in that it allows transport mechanisms to work independently of the technology they are based on [35].

Algorithm 1 describes the coding algorithm on the transmitter/server side. In many cases, the most critical factor for determining the pathway performance is RTT. Its estimation takes into account data transfer time, data lead time at the recipient, and SACK transfer rate. SACK may be sent on several paths in CMT, and varying delays on divergent routes lead to inaccurate RTT estimates. The coding subsystem is in charge of creating coded packets from original packets and keeping track of initial packets within the recipient buffer [36]. SACK (Selective Acknowledgment) is a method that rectifies this pattern when numerous segments are dropped. The data receiver can advise the sender about all portions that have arrived successfully using selective acknowledgments, requiring the sender to retransmit just the segments that have been lost [37]. The coding module generates a coded packet pk in the form of pk = ipi. The coded packet can be redundant or creative. The redundant packets contain linear equations containing the same unknown set as the preceding coded packet but with randomly chosen coefficients [38]. An innovative packet is one that is not the same as the last one that was coded. It has a different set of unknowns than the last one.

The client/receiver side decoding system process is described in Algorithm 2. When an innovative packet arrives from any of the paths, it is buffered, and the encoding equations are extracted from the incoming packets and applied to the decoding vector as a new row [39]. The recipient reconstructs and sends back the intended packets in the processing buffer to restore the initial video traffic for upper-layer applications [40].

## 5. Experimental Results and Outcomes

This section illustrates the simulation outcome that has been undergone using the Network Simulator 2. The flood surveillance network is assumed to have 50, 100, 150, 200, and 250 nodes. Three case studies have been applied in the experimental work to calculate packet loss, path failure, and transmission time, the rate of packet failure, end-to-end delay, and average throughput of different scheduling times [41]. The cases below have been used in a simulation environment to look at the CMT protocol for video surveillance and see how it works.

(i) Selecting the main pathway (P1) as the best option
  - If P1 fails, choose an AI (alternating path).
(ii) Case (b) Choosing P1 once more if A1 fails

Figure 3 shows the number of packets and time with respect to the primary and alternate paths. It is inferred that packet loss remains almost the same for both selections of paths P1 and A1. By utilizing sent and received packet tallies acquired from quality estimation packets, a strategy is utilized in which a packet check of value estimation packets sent from the sending test to the accepting test and a packet tally of value estimation packets sent from the getting test to the sending test are obtained [42]. At this point, the packet loss rate is found by following the method shown in [43].

(6) $$\begin{array}{c} \text{Packet loss }=\;100\text{\%}\frac{\left(\text{received packet }-\text{ sent packet}\right)}{\text{sent packet}}. \end{array}$$

Figure 4 shows the number of nodes vs. path failure, and it is understood that while choosing P1, there has been less packet loss by choosing A1.  Figure 5 demonstrates the quantity of network nodes vs. transmission time and it is shown that while choosing P1, there has been almost equal transmission time taken with different node numbers by choosing both A1 and P1. Usability validation is an important criterion that evaluates how different nodes interact with transmission time. It also refers to ways to make network design easier when it comes to the number of network nodes and the time it takes to send and receive data while it is being made.

It is clear from Figures 6, –7, and Fig 8 that the end-to-end delay, retransmission time, and throughput vary with small time variations even when P1 and A1 are chosen. Retransmission refers to resending packets that have been lost or destroyed via the network. Retransmission is a process employed by protocols to ensure that communication is dependable [38]. The networks are unreliable, and there is no guarantee that lost or damaged packets will be delayed or retransmitted. The transmission time in seconds can be obtained from the packet size as follows:

(7) $$\begin{array}{c} \text{Packet transmission time}=\frac{\text{Packet size}}{\text{Bit rate}}. \end{array}$$

End-to-end delay alludes toward the packet that consumes time to get communicated in the system from sender to receiver

(8) $$\begin{array}{c} \text{End}-\text{to}-\text{end delay}=\frac{N*L}{R}, \end{array}$$

where *N* = link, *L* = packet length, and *R* = transmission rate.

The efficiency of the proposed method can be evaluated by the average throughput, which refers to a whole payload in excess of the complete gathering separated as a result of the full time and total time being calculated by means of considering the variation in timestamps between the opening and final packet [35, 44].

From the experimental results, we have got an idea that by using video surveillance, the CMT algorithm suits well as far as reliability is concerned. Instantaneous databases, on-demand computing infrastructure, and storage are all made possible by cloud-based IoE. It also makes it easier to make apps that can analyze and process data from IoT devices [30, 45].

## 6. Discussion

The concurrent multipath transfer protocol has been implemented in the flood monitoring surveillance system by way of effective and efficient packet transfer during hostile environments during flooding in order to ensure the safe arrival of videos that have been captured by IoT enabled high definition cameras. The proposed protocol makes the video surveillance system more authenticated as far as reliability is concerned. The proposal also confirms that it has achieved better transmission time, throughput, and reduced packet loss comparatively. For the reason that the receiver buffer is only one of its kind, the lost packet has to be originated as rapidly as achievable for retransmission to keep away from all paths deteriorating into tender packets to higher layers merely for the abnormity of one path, which causes the jamming of the receiver's head-of-line blocking to restrict the pace of complete connection. In addition to that, permitting positioning of the missing packet between paths can cause a lost packet to be established immediately. The improved method of quick retransmit can reduce the number of avoidable quick retransmits, and the equal system between quick retransmit and timeout retransmit can resolve the issue that better speedy retransmits can be completed as a substitute for timeout retransmits.

## 7. Conclusion

This paper presented the urban flood high definition video surveillance system using a concurrent multipath transfer. Identifying the shortest path in the changeable surroundings at the same time as having fewer than three cases, namely, the main path as a perfect pathway, the main path failure, which shows the way to select the alternating pathway, and if the failure is on a substitute path, the ultimate aim of using concurrent paths by means of multihoming so as to reach the end point reliably without any delay or packet loss, has been achieved. The proposal suggests ways in which the amalgamation of IoT sensor techniques could enhance the quality of monitoring the flooding because of its reliable data transmission protocol. It also emphasizes the importance of real-time flood monitoring in the form of playing a significant role in flood modeling, mapping, and timely warning systems as well as the assessment of water level. In future work, concurrent multipath transfer under an instable network environment will be studied, and the retransmission time needs to be measured to further make the flood video surveillance system more reliable.

## Figures and Tables

**Figure 1:** Architecture view of the proposed system.

**Figure 2:** Communication flow of the proposed scheme.

**Figure 3:** Packet loss.

**Figure 4:** Path failure.

**Figure 5:** Time taken with different node numbers.

**Figure 6:** Packet loss rate and end to end delay.

**Figure 7:** Retransmission time with varying node numbers.

**Figure 8:** Average throughput.

**Algorithm 1:** At the server/transmitter side.

**Algorithm 2:** Decoding module at the receiver/client side.

## Data Availability

The data that support the findings of this study are available from the corresponding author on request.
